# Effects of Temperature and Precipitation on Breeding Migrations of Amphibian Species in Southeastern Norway

**DOI:** 10.1155/2016/3174316

**Published:** 2016-04-28

**Authors:** Børre K. Dervo, Kim Magnus Bærum, Jostein Skurdal, Jon Museth

**Affiliations:** Norwegian Institute of Nature Research (NINA), Human Dimension Department, Fakkelgården, 2624 Lillehammer, Norway

## Abstract

To reveal the effects of climate, a generalized linear mixed model was used to explore the variation in onset of spawning migration for the two newt species* T. cristatus* and* L. vulgaris* in southern Norway. Amphibians are highly influenced by the physical environment, such as temperature and rainfall. The first migrating newts were observed subsequently to the three first consecutive days with mean temperature close to or above 4°C. Further, migration of* L. vulgaris* was facilitated at lower temperatures compared to* T. cristatus*, but the migration was dependent on higher precipitation levels. Northern populations of* T. cristatus* and* L. vulgaris* may already benefit from a warmer climate due to increased recruitment and juvenile survival. However, an offset in the migration phenology due to climate change might further alter the recruitment and survival rates with either positive or negative outcome. Thus, variations in migration phenology for newts due to climate change may have implications for management and protection status in many systems. In a general context, we should increase emphasis on protecting newts and support increased populations and distribution.

## 1. Introduction

Amphibian populations are declining at an alarming pace in many parts of the world [1–6]. As amphibians, and ectotherms in general, are highly influenced by the physical environment, a number of these declines could be directly or indirectly linked to climate change [7–9]. In general, global meta-analyses document significant range shifts for different species averaging 6.1 km per decade towards the poles and significant mean advancement of spring events by 2.3 days per decade [10]. Precipitation level and temperature especially are expected to be affected by climate change, and in the Northern Hemisphere a decadal increase in temperature of 0.7–1.0% and a decadal increase in precipitation 10−20% are observed [11, 12].

These are key climate components acting directly on processes important for the population dynamics, especially for amphibians. As the skin is highly permeable, amphibians are sensitive to moisture conditions [13, 14]. Temperature acts as a controlling agent for many physiological processes including rates of oxygen uptake, heart rate, locomotion, water balance, digestion, developmental rate, sex determination, and immune function [15]. Further, the gametogenesis and growth rates of larval and postmetamorphic individuals are also temperature dependent [16, 17]. Additionally, climatic factors may affect important processes such as breeding phenology, migrations, and mating [16, 18–20].

It is perhaps surprising that even though the effect of single environmental variables on different physiological aspects might be well represented in the literature, population declines as a consequence of climate change are not always well understood [7, 8]. However, the natural environment is rarely defined by single variables, but rather a range of potential interactions that paints a more complex feedback picture of climate change for ectotherms [21–23]. There exists some knowledge in the literature on how changes in single components of the environment (e.g., temperature) might alter the phenology of amphibians (see, e.g., [19, 24, 25]); however empirical studies on the combined effect of multiple interacting environmental variables in the wild are rare. Nonetheless, such information is vital for future understanding of climate change, conservation efforts, and management decisions for amphibians [26].

In this study we focused on two amphibian species,* Triturus cristatus* (Laurenti, 1768) and* Lissotriton vulgaris* (Linnaeus, 1758).* T. cristatus* populations are declining in many European countries [27–29], whereas* L. vulgaris* are still widespread and locally abundant [30–33]. Both species are semiaquatic with overlapping timing of daily and seasonal activities and they often inhabit the same landscapes and water bodies [30, 34–36]. The interspecific interactions are expected to be weak due to differences in their feeding habits, microhabitats, and diel activity pattern [30, 31].* T. cristatus *depend more on water depth and aquatic vegetation than* L. vulgaris, *but both species are believed to be affected by the same ecological processes [37]. Both species have their northern limit of distribution in Scandinavia.* L. vulgaris* are more widespread than* T. cristatus* in Norway [38]. Climatic regimes influence species distribution, often through species-specific physiological thresholds of temperature and precipitation tolerance. The migration between breeding and hibernation areas in spring and autumn is a critical phase with increased mortality, and possible shifts in this migration event due to climate change could thus have consequences at a population level.

Normally newts initiate their migration in spring at the end of frost periods with increasing temperatures and when stimulated by rainfall [39, 40]. Here we wanted to explore variations in phenology, that is, onset of spawning migration, as a function of these two fundamental environmental factors which are affected by climate change [12]. Further, we discuss how expected future climate scenarios might influence the breeding migration of newts and how an expected shift to earlier spawning migration might influence population development of the two species.

## 2. Material and Methods

The study pond and surrounding area in Lier municipality, Buskerud County, southeastern Norway (UTM WGS84 33N 0236699 33S 6630232), are severely impacted by human use and dominated by agriculture, private homes, and infrastructure (Figure 1). The breeding pond Lahelldammen (30 m asl) has an area of 6,050 m^2^, max depth of 4 m, and a volume of 13,000 m^3^. Mean annual air temperature is 5.0°C and mean annual precipitation is 860 mm. Mean monthly air temperatures in March, April, and May are −1.0, 3.9, and 10.1°C, respectively (eKlima.no). The 0.392 km^2^ area within a 300 m distance from the pond is used for agriculture (33%), roads (6%), and housing (17%) (GIS-based analysis of FKB-map from the Norwegian Mapping Authority). Forest and nature-like areas constitute 44% of the area. Only 29% of the area is easily accessible for newts due to two roads (Røykenveien and Grimsrudveien) with high motor traffic and a nearby river. Approximately 10% of the area is characterized as “well suited” newt habitat. The pond is a breeding site for* T. cristatus, L. vulgaris*,* Rana temporaria*,and* Bufo bufo*. The local road around Lahelldammen is used by only a few cars every day and is therefore suitable for observing newt crossings. In a mark-recapture experiment, we found that approximately 25% of the population of* T. cristatus* hibernated in the area inside the road and furthermore the study revealed that approximately 40% of the newts crossing the road were observed by our road counts (Dervo unpubl.). Based on the mark-recapture study, the average annual* T. cristatus* population was estimated (Chapman estimator) to be 1 156 (95% CI = 738–1 573) mature individuals for the years 2012–2015. For* L. vulgaris*, no mark-recapture data existed for population estimates; however based on the counts during migration and the ratio between* T. cristatus* and* L. vulgaris* captured,* L. vulgaris* population was estimated to include approximately 7 600 mature individuals.

Newt spring migration patterns were recorded every day in five consecutive years (2010–2014) from February to May. The exceptions were days with very unfavorable conditions for migration (e.g., freezing temperatures), where no recordings were conducted. The newts were counted using a flashlight at night [41, 42] on a 501 m long and 6 m wide paved road, encircling the breeding pond Lahelldammen. For each individual count, time, position, species, and sex were registered. The number of observation rounds each night ranged from 0 to 15 starting approximately 1 hour after sunset. When conditions were unfavorable, that is, cold weather and more than a week since the last rainfall, we skipped the observations. When the numbers of newts observed were low (<5 ind.) only two observation rounds were performed. Overall, 1 460 great crested newts and 8 234 smooth newts were observed during 163 observation days and 648 observation rounds (Table 1). On selected days we made observations to find the time when the first newts crossed the road. Temperature and precipitation data are from the Norwegian Meteorological Institute's weather station at Berskog-Drammen (8 m asl) located 8 km from the study area (eKlima.no). Temperature and light conditions were measured by a HOBO Pendant Temperature Data Logger (±0.53°C and ±2.5% FS for light) (http://www.onsetcomp.com/products/data-loggers/ua-001-64) when the first crossing newts were observed.

## 3. Statistical Analyses

All statistical analyses were done in the statistical software R, version 3.01 [43], utilizing the lme4 package [44]. We used a generalized linear mixed model approach to explore the count of newts per observation round as functions of temperature and precipitation and the interaction between these two explanatory variables. Specifically the newt count was assumed to be strictly proportional to the numbers of observation rounds (i.e., using numbers of observation rounds as an offset). Further, we assumed the response variable (i.e., newt counts) to have a Poisson distribution. We constructed multiple candidate models, for both* T. cristatus *and* L. vulgaris*, that included different variations of the variables in focus (Table 2) as fixed effects. We also included year and year specific proportion of newts that already migrated (divided in 5 quartile groups) as random intercept terms. The proportion of newts that already migrated each year was included to account for the reduced migration potential in the population as the proportion increased towards one.

The different candidate models exploring numbers of migrators for each migration potential group thus represented either of the following models:

(1) Yij=β0ij+β1ijxTij+β2ijxPij+β3ijxTijxPij+ai+εij,Yij=β0ij+β1ijxTij+β2ijxPij+ai+εij,Yij=β0ij+β1ijxTij+ai+εij,Yij=β0ij+β1ijxPij+ai+εij,

where *x*_*T*_ and *x*_*P*_ each represent one of the temperature and precipitation candidate variables (Table 2), respectively, for year *i* and grouped proportion of newts that migrated *j*. *β*s represent coefficients under estimation, *a*_*i*_ is the random year intercept, and *ε*_*ij*_ is the random residual variation.

As we might expect a nonlinear response of migration pattern to both precipitation and temperature, polynomials of degrees 2 and 3 were also included in some candidate models. The rationality of also exploring polynomials of degree 3 was to explore a smoother nonlinear relationship, compared to the assumption of a stricter parabola shaped relationship produced by the polynomial of degree 2. The most supported model was selected based on weighted AICc-values [45] derived from the AICcmodavg package [46].

## 4. Results

The spring migration period and number of migrators of both* T. cristatus* and* L. vulgaris* varied between years (Figure 2). In general, the first observations of migrating newts were done subsequently to the three first consecutive days of the year with mean temperature close to or above 4°C (Table 3). This occurred as early as February 27 in 2014 and as late as April 11 in 2013 for* T. cristatus* (Table 1, Figure 2).* L. vulgaris* had its earliest spring migration on March 7 in 2014 and as late as April 11 in 2013 (Table 1). The migrations were initiated in the evening when the light conditions diminished to roughly 5 lux, that is, around 8 PM at the beginning of the migration period in February and at 10 PM at the end of May. Most individuals migrated during the first three hours and the migrations usually peaked around midnight (Figure 3). Migrations at temperatures below zero were registered only once whereas most migrating newts (94%) were observed at temperatures above 1.5°C.

For* T. cristatus*, the most supported model describing the migration pattern included an interaction term of daily mean temperature and a third-degree polynomial of the accumulated day specific precipitation (Tables 4 and 5). This model (approximated conditional *R* ^2^ = 0.12) predicted an almost exponential increase in numbers of migrators starting at mean daily temperatures between 13 and 14°C. The positive temperature effect was however very much dependent on the precipitation levels, where accumulated daily precipitation at approximately 6 mm seemed to facilitate the highest migration rates (Figure 4). Consequently, increasing or decreasing precipitations levels above or below ~6 mm resulted in fewer migrators. This trend was especially apparent at higher temperatures.

The most supported model of migration pattern for* L. vulgaris* included an interaction term of the mean temperature over the last 3 days and a third-degree polynomial of the accumulated day specific precipitation (Tables 5 and 6). The model (approximated conditional *R* ^2^ = 0.13) predicted a positive response of temperature. As for* T. cristatus*, this response was also very dependent on the precipitation level (Figure 5). In general, migration of* L. vulgaris* was facilitated at lower temperatures compared to* T. cristatus*, but the migration was dependent on higher precipitation levels. Numbers of smooth newt migrators were generally low when daily precipitation was below 11-12 mm at all temperatures but increased when the daily precipitation was in the range from ~11 to ~17 mm. The latter trend was especially apparent at higher temperatures. Precipitation levels above ~17 mm generally resulted in decreasing numbers of migrators; however these high precipitation levels facilitated migration at low temperatures (i.e., <10°C). Analysis did not reveal any significant differences between females and males in migration pattern.

## 5. Discussion

We found interspecific variation in spawning migration pattern between the two amphibian species,* T. cristatus *and* L. vulgaris*, as functions of temperature and precipitation. Both species initiated their spring migration subsequently to the first-three-day period with mean temperature at approximately 4°C. Interannual variation in climate conditions resulted in a variance of 43 days for the initiation of the migration during the study period. Precipitation was important for the migration pattern of both species. For* L. vulgaris*, numbers of migrators increased at lower temperatures but were dependent on higher precipitation levels as compared to* T. cristatus*. Further, the most supported model for* L. vulgaris* included mean temperature during the last 72 hours instead of mean temperature of the last 24 hours, as for* T. cristatus*. This could indicate that* L. vulgaris* are dependent on more stable temperatures compared to* T. cristatus *in order to sustain high numbers of migrators. In late springs with cold weather the migration period was short, that is, 23 days, compared to early and warm springs, that is, 40 days. In general, the migration periods in these northern populations of newts were shorter compared to what was found for populations further south [19, 40, 47, 48]. However, this difference was less in warm springs with early migrations.

The observed decline in amphibian populations may directly or indirectly be linked to climate change as precipitation and temperature are key climate components acting directly on processes important for the population dynamics for amphibians [9, 16, 18, 19, 24, 25]. The migration phenology of both newt species in our study was clearly affected by the combined effect of both temperature and precipitation levels, with an overall trend of earlier onset of breeding migration with increasing temperatures. Our predicted change in reproductive timing because of global warming concurs with other studies on amphibians (e.g., [49, 50]) as well as species from other taxa (e.g., [51–54]). Very few studies, however, focus on the combined effect of multiple climate components. Given the strong support for the interactive effect for both precipitation and temperature on the migration phenology of the amphibians in our study, we urge that both components should be considered in future studies of climate effects. Though the population effects of climate change are not straightforward as multiple climate components, life history traits and environmental properties interact to alter the population effects depending on settings (e.g., [21, 55, 56]). The ecological consequences of an earlier spring may be positive for amphibian populations that live on the northern border of their range [9, 57]. Early migration and breeding might increase the time available for juveniles to feed before their first winter, thus providing increased recruitment [58]. Numerous field studies have supported the idea that juveniles are more likely to disperse to new sites than adults and, therefore, likely constitute the dispersal stage for pond-breeding species [59–61]. Increased recruitment might facilitate colonization of new localities and increase the poleward distribution [57]. Earlier spring might also reduce predation risk before the first reproduction and increasing breeding opportunity [62].

Northern populations of* T. cristatus* and* L. vulgaris* may already benefit from a warmer climate due to increased recruitment and juvenile survival whereas population may decline in other areas due to the combination of climate change and the local climate. In our study area, the winters are cold, snow may accumulate in winter providing improved hibernation condition (e.g., better isolation) for newts, and combined with a longer growth period this will enhance survival. Increased winter precipitation in Southern England however had the adverse effect as survival was reduced [29].

## 6. Conclusions

The models reveal interspecific variation in spawning migration pattern between the two amphibian species,* T. cristatus *and* L. vulgaris*, as functions of temperature and precipitation. Both climate components are thus important to include for future understanding of climate effects on amphibians in general. Northern populations of* T. cristatus *and* L. vulgaris *may already benefit from a warmer climate due to increased recruitment and juvenile survival. Both species have increased in numbers and distribution in Norway the last decade [38, 63]. This may influence management and Red List status in northern regions and reduce the protection regime. However, in a general context we should increase emphasis on protecting newts and support increased populations and distribution as climate change may have adverse effects on populations further south.

## Figures and Tables

**Figure 1:** Map of the pond Lahelldammen (UTM WGS84 33N 0236699 33S 6630232) in southeastern Norway with the route for observation (Lahelldammen road, black line) and areas which are difficult to access are hatched.

**Figure 2:** The daily numbers of observed spring migrators of great crested newt* T. cristatus *(open bars) and smooth newt* L. vulgaris* (black bars) at Lahelldammen in the period 2010 (a) to 2014 (e).

**Figure 3:** Time of the day for observations of migrating* T. cristatus *(open bars, April 7-8, 2014) and* L. vulgaris *(black bars, April 6-7) at Lahelldammen in 2014.

**Figure 4:** Contour plot of predicted numbers of migrating* T. cristatus* per observation unit, as a function of daily mean temperatures in °C (*x*-axis) and accumulated daily precipitation in mm (*y*-axis). Maximum numbers of migrators are restricted to 20 individuals in the plot to ease visualization.

**Figure 5:** Contour plot of predicted numbers of migrating* L. vulgaris* per observation unit, as a function of daily mean temperatures (°C) over the three last days since the specific observation (*x*-axis) and accumulated daily precipitation in mm (*y*-axis). Only every third contour is shown in the plot to ease visualization.

**Table 1:** Number of observed individuals of *T. cristatus* (Tc) and *L. vulgaris *(Lv), the first and last day of observation, the number of observation days, and the number of observation rounds for the period 2010 to 2014.

Year	2010	2011	2012	2013	2014
Number of ind. Tc	200	170	396	326	368
Number of ind. Lv	1240	1088	2663	2066	1177
First obs. day Tc	Apr. 7	Apr. 3	Mars 17	Apr. 11	Feb. 27
Last obs. day Tc	May 19	Apr. 25	May 11	May 7	May 9
First obs. day Lv	Apr. 7	Apr. 4	Mars 17	Apr. 11	Mars 7
Last obs. day Lv	May 19	Apr. 29	May 11	May 7	May 9
Number of obs. days	34	27	40	23	39^*∗*^
Number of obs. rounds	109	79	200	139	121

^*∗*^On April 7 no observations of *L. vulgaris* were made because of too many *T. cristatus*.

**Table 2:** Variables considered in the fixed effect structure of the various candidate models for describing newt migration phenology pattern as a function of temperature and precipitation.

Candidate variables	Description
Accumulated temperature total (AT)	Degree days of daily mean temperatures in °C after 1 observation of migrating newts
Accumulated temperature 3 (AT3)	Degree days of daily mean temperatures in °C over the 3 last days since each respective migration observation
Accumulated temperature 5 (AT5)	Degree days of daily mean temperatures in °C over the 5 last days since each respective migration observation
Mean temperature (MT)	Mean air temperature of the last 24 hours since each respective observation
Mean temperature 3 (MT3)	Mean air temperature of the last 72 hours since each respective observation
Mean temperature 5 (MT5)	Mean air temperature of the last 120 hours since each respective observation
Precipitation (P)	Sum of precipitation values in mm during the last 24 hours since each respective observation
Precipitation 3 (P3)	Sum of precipitation values in mm during the last 72 hours since each respective observation
Precipitation 5 (P5)	Sum of precipitation values in mm during the last 120 hours since each respective observation

**Table 3:** Temperature statistics and specific dates for the first day of observation of *T. cristatus* from 2010 to 2014. Precipitation levels are not included in the table as they were all 0–0.1 mm. Detailed variable descriptions are provided in Table 2. First observations of *L. vulgaris* coincided with *T. cristatus* for all years, except for 2011 and 2014, where the first observations were registered one and eight days later, respectively.

Date	MT/AT	MT3	MT5	AT3	AT5
April 7, 2010	5.2	4.4	3.9	13.1	19.7
April 3, 2011	4.8	4.1	2.4	12.4	12
March 17, 2012	5.2	3.8	5.5	11.3	27.3
April 14, 2013	2.6	6.3	7.5	18.9	37.6
February 27, 2014	3.8	3.5	4.3	10.5	21.5

**Table 4:** Parameter estimates for the most supported model exploring effects of temperature and precipitation on the breeding migration pattern of *T. cristatus*.

Parameters	Estimate	Std. error	*z*-value	Pr > *z*
Intercept	−7.73	1.54	−5.01	<0.001
MT	0.13	0.03	4.99	<0.001
P	−6.82	1.18	−5.77	<0.001
P^2^	20.17	1.08	18.61	<0.001
P^3^	−4.24	1.14	−3.70	<0.001
MT × P	1.81	0.16	11.04	<0.001
MT × P^2^	−2.44	0.14	−16.93	<0.001
MT × P^3^	1.87	0.20	9.45	<0.001

**Table 5:** Model selection table based on AIC-values for the three most supported mixed models exploring breeding migration pattern for *T. cristatus* (upper) and *L. vulgaris* (lower).

Model	*K*	AICc	ΔAIC	AIC-weight
*Great crested newt*				
MT × P^3^	10	5518.45	0	1
MT × P3^3^	10	5718.74	200.29	0
MT^3^ × P	10	5824.60	306.16	0

*Smooth newt*				
MT3 × P^3^	10	34887.85	0	1
MT × P^3^	10	35471.67	583.82	0
AT × P^3^	10	36089.54	1201.69	0

**Table 6:** Parameter estimates for the most supported model exploring effects of temperature and precipitation on the breeding migration pattern of *L. vulgaris*.

Parameters	Estimate	Std. error	*z*-value	Pr > *z*
Intercept	−1.21	1.24	−0.97	0.332
MT3	−0.29	0.01	−26.12	<0.001
P	3.84	0.35	11.06	<0.001
P^2^	4.56	0.41	11.19	<0.001
P^3^	11.94	0.30	40.19	<0.001
MT3 × P	0.94	0.05	17.34	<0.001
MT3 × P^2^	−0.36	0.07	−5.01	<0.001
MT3 × P^3^	−1.29	0.05	−25.54	<0.001

## References

[1] Beebee T. J. C., Griffiths R. A. (2005). The amphibian decline crisis: a watershed for conservation biology?. *Biological Conservation*.

[2] Blaustein A. R., Wake D. B. (1995). The puzzle of declining amphibian populations. *Scientific American*.

[3] Hof C., Araújo M. B., Jetz W., Rahbek C. (2011). Additive threats from pathogens, climate and land-use change for global amphibian diversity. *Nature*.

[4] Stuart S. N., Chanson J. S., Cox N. A. (2004). Status and trends of amphibian declines and extinctions worldwide. *Science*.

[5] Houlahan J. E., Fidlay C. S., Schmidt B. R., Meyer A. H., Kuzmin S. L. (2000). Quantitative evidence for global amphibian population declines. *Nature*.

[6] Zuiderwijk A. (1990). Sexual strategies in the newts *Triturus cristatus* and *Triturus marmoratus*. *Bijdragen tot de Dierkunde*.

[7] Carey C., Alexander M. A. (2003). Climate change and amphibian declines: is there a link?. *Diversity and Distributions*.

[8] Parmesan C. (2006). Ecological and evolutionary responses to recent climate change. *Annual Review of Ecology, Evolution, and Systematics*.

[9] Blaustein A. R., Walls S. C., Bancroft B. A., Lawler J. J., Searle C. L., Gervasi S. S. (2010). Direct and indirect effects of climate change on amphibian populations. *Diversity*.

[10] Parmesan C., Yohe G. (2003). A globally coherent fingerprint of climate change impacts across natural systems. *Nature*.

[11] Walther G.-R., Post E., Convey P. (2002). Ecological responses to recent climate change. *Nature*.

[12] IPCC (2013). *Climate Change 2013: The Physical Science Basis*.

[13] Duellman W. E., Trueb L. (1986). *Biology of Amphibians*.

[14] Hillyard S. D. (1999). Behavioral, molecular and integrative mechanisms of amphibian osmoregulation. *Journal of Experimental Zoology*.

[15] Feder M. E., Burggren W. W. (1992). *Environmental Physiology of the Amphibians*.

[16] Beebee T. J. C. (1995). Amphibian breeding and climate. *Nature*.

[17] Carey C., Corn P. S., Jones M. S., Livo L. J., Muths E., Loeffler C. W. (2005). Factors limiting the recovery of boreal toads (*Bufo b. boreas*). *Amphibian Declines: The Conservation Status of United States Species*.

[18] Blaustein A. R., Belden L. K., Olson D. H., Green D. M., Root T. L., Kiesecker J. M. (2001). Amphibian breeding and climate change. *Conservation Biology*.

[19] Chadwick E. A., Slater F. M., Ormerod S. J. (2006). Inter- and intraspecific differences in climatically mediated phenological change in coexisting *Triturus* species. *Global Change Biology*.

[20] Forchhammer M. C., Post E., Stenseth N. C. (1998). Breeding phenology and climatet. *Nature*.

[21] Bærum K. M., Haugen T. O., Kiffney P., Moland Olsen E., Vøllestad L. A. (2013). Interacting effects of temperature and density on individual growth performance in a wild population of brown trout. *Freshwater Biology*.

[22] Crozier L. G., Zabel R. W., Hockersmith E. E., Achord S. (2010). Interacting effects of density and temperature on body size in multiple populations of Chinook salmon. *Journal of Animal Ecology*.

[23] McCain C. M., Colwell R. K. (2011). Assessing the threat to montane biodiversity from discordant shifts in temperature and precipitation in a changing climate. *Ecology Letters*.

[24] Kusano T., Inoue M. (2008). Long-term trends toward earlier breeding of Japanese amphibians. *Journal of Herpetology*.

[25] Todd B. D., Scott D. E., Pechmann J. H. K., Whitfield Gibbons J. (2011). Climate change correlates with rapid delays and advancements in reproductive timing in an amphibian community. *Proceedings of the Royal Society B: Biological Sciences*.

[26] Clusella-Trullas S., Blackburn T. M., Chown S. L. (2011). Climatic predictors of temperature performance curve parameters in ectotherms imply complex responses to climate change. *The American Naturalist*.

[27] Edgar P., Bird D. R. (2006). *Action Plan for the Conservation of the Crested Newt Triturus cristatus Species Complex in Europe*.

[28] Denoël M. (2012). Newt decline in Western Europe: highlights from relative distribution changes within guilds. *Biodiversity and Conservation*.

[29] Griffiths R. A., Sewell D., McCrea R. S. (2010). Dynamics of a declining amphibian metapopulation: survival, dispersal and the impact of climate. *Biological Conservation*.

[30] Griffiths R., Mylotte V. (1987). Microhabitat selection and feeding relations of smooth and warty newts, *Triturus vulgaris* and *T. cristatus*, at an upland pond in mid-Wales. *Ecography*.

[31] Dolmen D. (1988). Coexistence and niche segregation in the newts *Triturus vulgaris* (L.) and *T. cristatus* (Laurenti). *Amphibia-Reptilia*.

[32] Fog K., Schmedes A., Rosenørn de Lasson D. (1997). *Nordens Padder Og Krybdyr*.

[33] Rannap R., Lohmus A., Linnamägi M. (2012). Geographic variation in habitat requirements of two coexisting newt species in Europe. *Acta Zoologica Academiae Scientiarum Hungaricae*.

[34] Zuiderwijk A., RočekCharles Z. (1986). Competition, coexistence and climatic conditions: influence on the distribution of the warty newt, *Triturus cristatus*. *Western Europe. Studies in Herpetology*.

[35] Skei J. K., Dolmen D., Rønning L., Ringsby T. H. (2006). Habitat use during the aquatic phase of the newts *Triturus vulgaris* (L.) and *T. cristatus* (Laurenti) in central Norway: proposition for a conservation and monitoring area. *Amphibia-Reptilia*.

[36] Van Buskirk J. (2007). Body size, competitive interactions, and the local distribution of *Triturus* newts. *Journal of Animal Ecology*.

[37] Denoël M., Perez A., Cornet Y., Ficetola G. F. (2013). Similar local and landscape processes affect both a common and a rare newt species. *PLoS ONE*.

[38] ADB (2015). *Species Map Service 1.6*.

[39] Malmgren J. C. *Åtgärdsprogram för Bevarande av Större Vattensalamander Och Dess Livsmiljöer (Triturus cristatus)*.

[40] Harrison J., Gittins S., Slater F. (1983). The breeding migration of smooth and palmate newts (Triturus vulgaris and T. helveticus) at a pond in mid Wales. *Journal of Zoology*.

[41] Cooke A. S. (1995). A comparison of survey methods for crested newts (*Triturus cristatus*) and night counts at a secure site, 1983-1993. *Herpetological Journal*.

[42] Kupfer A. (1996). *Untersuchungen zur populationsökologie, phänologie und ausbreitung des kammolches triturus cristatus (Laurenti 1768) in einem agrarraum des drachenfelser ländchens bei Bonn [Diplomarbeit]*.

[43] R Core Team R. (2014). *R: A Language and Environment for Statistical Computing*.

[44] Bates D., Maechler M., Bolker B., Walker S. (2014). *Linear Mixed-Effects Models Using Eigen and S4*.

[45] Burnham K. P., Anderson D. R. (2002). *Model Selection and Multimodel Inference: A Practical Information-theoretic Approach*.

[46] Mazerolle M. J. Model selection and multimodel inference based on (Q)AIC(c).

[47] Jehle R., Arntzen J. W. (2000). Post-breeding migrations of newts (*Triturus cristatus* and *T. marmoratus*) with contrasting ecological requirements. *Journal of Zoology*.

[48] Verrell P., Halliday T. (1985). The population dynamics of the crested newt *Triturus cristatus* at a pond in southern England. *Holarctic Ecology*.

[49] Todd B. D., Scott D. E., Pechmann J. H. K., Gibbons J. W. (2011). Climate change correlates with rapid delays and advancements in reproductive timing in an amphibian community. *Proceedings of the Royal Society B: Biological Sciences*.

[50] Klaus S. P., Lougheed S. C. (2013). Changes in breeding phenology of eastern Ontario frogs over four decades. *Ecology and Evolution*.

[51] Both C., Visser M. E. (2005). The effect of climate change on the correlation between avian life-history traits. *Global Change Biology*.

[52] Cotton P. A. (2003). Avian migration phenology and global climate change. *Proceedings of the National Academy of Sciences of the United States of America*.

[53] Van Buskirk J., Mulvihill R. S., Leberman R. C. (2009). Variable shifts in spring and autumn migration phenology in North American songbirds associated with climate change. *Global Change Biology*.

[54] Végvári Z., Bókony V., Barta Z., Kovács G. (2010). Life history predicts advancement of avian spring migration in response to climate change. *Global Change Biology*.

[55] Sæther B.-E., Tufto J., Engen S., Jerstad K., Røstad O. W., Skåtan J. E. (2000). Population dynamical consequences of climate change for a small temperate songbird. *Science*.

[56] Vindenes Y., Edeline E., Ohlberger J. (2014). Effects of climate change on trait-based dynamics of a top predator in freshwater ecosystems. *The American Naturalist*.

[57] Araújo M. B., Thuiller W., Pearson R. G. (2006). Climate warming and the decline of amphibians and reptiles in Europe. *Journal of Biogeography*.

[58] Reading C. J., Clarke R. T. (1999). Impacts of climate and density on the duration of the tadpole stage of the common toad Bufo bufo. *Oecologia*.

[59] Kupfer A., Kneitz S. (2000). Population ecology of the great crested newt (*Triturus cristatus*) in an agricultural landscape: dynamics, pond fidelity and dispersal. *Herpetological Journal*.

[60] Breden F. (1987). The effect of post-metamorphic dispersal on the population genetic structure of Fowler's toad, *Bufo woodhousei fowleri*. *Copeia*.

[61] Berven K. A., Grudzien T. A. (1990). Dispersal in the wood frog (*Rana sylvatica*): implications for genetic population structure. *Evolution*.

[62] Berven K. A. (1990). Factors affecting population fluctuations in larval and adult stages of the wood frog (*Rana sylvatica*). *Ecology*.

[63] DN Handlingsplan for stor salamander *Triturus cristatus*. Direktoratet for naturforvaltning. *DN-Rapport*.

